# Immunization with H7-HCP-Tir-Intimin Significantly Reduces Colonization and Shedding of *Escherichia coli* O157:H7 in Goats

**DOI:** 10.1371/journal.pone.0091632

**Published:** 2014-03-14

**Authors:** Xuehan Zhang, Zhengyu Yu, Shuping Zhang, Kongwang He

**Affiliations:** 1 Institute of Veterinary Medicine, Jiangsu Academy of Agricultural Sciences, Nanjing, P. R. China; 2 Key Laboratory of Engineering Research of Veterinary Bio-products of Agricultural Ministry, Nanjing, P. R. China; 3 National Center for Engineering Research of Veterinary Bio-products, Nanjing, P. R. China; 4 Jiangsu Co-innovation Center for Prevention and Control of Important Animal Infectious Diseases and Zoonoses, Yangzhou, P. R. China; 5 Department of Veterinary Pathobiology, College of Veterinary Medicine, University of Missouri, Columbia, Missouri, United States of America; University of Padova, Medical School, Italy

## Abstract

Enterohemorrhagic *Escherichia coli* (EHEC) O157:H7 is the causative agent of hemorrhagic colitis and hemolytic uremic syndrome in humans. However, the bacterium can colonize the intestines of ruminants without causing clinical signs. EHEC O157:H7 needs flagella (H7) and hemorrhagic coli pili (HCP) to adhere to epithelial cells. Then the bacterium uses the translocated intimin receptor (Tir) and an outer membrane adhesion (Intimin) protein to colonize hosts. This leads to the attachment and effacement of (A/E) lesions. A tetravalent recombinant vaccine (H7-HCP-Tir-Intimin) composed of immunologically important portions of H7, HCP, Tir and Intimin proteins was constructed and its efficacy was evaluated using a caprine model. The results showed that the recombinant vaccine induced strong humoral and mucosal immune responses and protected the subjects from live challenges with EHEC O157:H7 86-24 stain. After a second immunization, the average IgG titer peaked at 7.2×10^5^. Five days after challenge, *E. coli* O157:H7 was no longer detectable in the feces of vaccinated goats, but naïve goats shed the bacterium throughout the course of the challenge. Cultures of intestinal tissues showed that vaccination of goats with H7-HCP-Tir-Intimin reduced the amount of intestinal colonization by EHEC O157:H7 effectively. Recombinant H7-HCP-Tir-Intimin protein is an excellent vaccine candidate. Data from the present study warrant further efficacy studies aimed at reducing EHEC O157:H7 load on farms and the contamination of carcasses by this zoonotic pathogen.

## Introduction

Enterohemorrhagic *Escherichia coli* (EHEC) O157:H7 is a zoonotic enteric pathogen associated with hemorrhagic colitis (HC) and hemolytic uremic syndrome (HUS) in humans. Ruminants are the main reservoir of *E. coli* O157:H7 which usually colonizes the intestinal tract without causing clinical signs [1]. Infected animals can shed the bacteria in their feces, so becoming direct or indirect sources of human infections via contaminated food or water [**1]**–[**2**]. For this reason, EHEC O157:H7 control in ruminants merits more attention.

Reductions in the number of EHECO157:H7 infection in cattle and in feces excreted by asymptomatic shedders can significantly decrease the risk of human exposure to this pathogen [**3**]. Vaccination of cattle has been proposed as a pre-harvest intervention strategy to reduce the amount of EHEC O157:H7 transmission from cattle. Inoculations of cattle with type III secreted proteins decreases fecal shedding of *E. coli* O157:H7 [**4**]. Vaccines based on siderophore receptors and porin (SRP) can reduce the burden of *E. coli* O157:H7 on cattle [**5**]. Systemic vaccination of cattle with γ-intimin C280 and EspB proteins decreases the fecal shedding of *E. coli* O157:H7 [**6**]. Immunization of cattle with a combination of purified intimin-531, EspA and translocated intimin receptor (Tir) significantly reduces shedding of *E. coli* O157:H7 after oral challenge [**7**]. Vaccination with *E. coli* O157 bacterial ghosts was found to provide protection in a bovine experimental model [**8**]. These vaccine formulations may become important tools in the control of EHEC O157:H7 transmission between animals and from animals to humans.

The versatile virulence factors contributing to *E. coli* O157:H7colonization of the gastrointestinal epithelium include outer membrane proteins, type III secretion system (T3SS) proteins, flagella, and pili. These proteins are often chosen to construct recombinant vaccines. Among them, intimin (*eae* gene) and Tir (*tir* gene) are key colonization factors, which paly significant roles in *E. coli* O157:H7attachment to host epithelium [**4]**–[**7**]. H7 flagellin encoded by the *fliC* gene is another interesting virulence factor. It reduces the rate of colonization but not that of overall bacterial shedding [**9**]. Hemorrhagic coli pili (HCP) are long bundles of type IV pili (TFP). These also contribute to bacterial colonization, virulence, and transmission of *E. coli* O157:H7 [**10]**–[**12**].

Because intimin, Tir, H7 flagellin, and HCP are critical to many of the stages of intestinal colonization by *E. coli* O157:H7, and recombinant subunit vaccines consisting of these proteins may hold the key to successful pre-harvest intervention of *E. coli* O157:H7. To test this hypothesis, a multivalent H7-HCP-Tir-Intimin protein was constructed and expressed for use as a vaccine candidate. A caprine model involving two-month-old goats was established to evaluate the effectiveness of H7-HCP-Tir-Intimin vaccine in the prevention of the colonization and spreading of *E. coli* O157:H7.

## Materials and Methods

### Ethics Statement

The care of laboratory animals and animal experimentation were performed in compliance with the Jiangsu Administration Guidelines for the Use of Experimental Animals. This study and all procedures were approved by the Animal Ethics Committee of Jiangsu Institute of Veterinary Medicine (SYXK20111101).

### Bacterial Strains, Plasmids and Media

The bacterial strains and plasmids used in this study are listed in **Table 1**. *E. coli* O157:H7 86-24 is a well-characterized Shiga-toxin-producing strain. Plasmid Pcold I and pET32 were acquired from TaKaRa Corp. Bacteria are grown in Luria-Bertani (LB) broth and on LB agar (Oxoid) supplemented with 100 µg/mL of ampicillin as needed for selection of recombinant plasmids. *E. coli* O157:H7 was recovered from a freezer and cultured in brain-heart infusion (BHI) broth.

**Table 1:** Bacterial strains and plasmids used in this study.

Strain or plasmid	Description	Source
*E. coli* strain		
O157:H786-24	Produce stx1and stx2	Current lab
BL21 (DE3)	Host for expressing recombinant plasmid	Transgen
Vectors		
Pcold I	*E. coli* expression vector	Takara
pET32a	*E. coli* expression vector	Novagen
Recombinant plasmids		
pET32-*fliC*	pET32 carrying 538–1483 bp of *fliC*	Current lab
pET32-*hcp*A	pET32 carrying 19–441 bp of *hcp*A	Current lab
pET32-*tir*	pET32 carrying 775–1083 bp of *tir*	Current lab
pET32-*eae*	pET32 carrying 1995–2805 bp of *eae*	Current lab
Pcold I-*fliC-hcpA*-*tir*-*eae*	*fliC-hcpA*-linker-*tir*-linker-*eae* cloned into Pcold I	Present study

### Plasmid Construction

Fragments of *fliC*, *hcpA*, *tir*, and *eae* were amplified by PCR from DNA isolated from *E. coli* O157:H7 86-24 strain with primers *fliC*-P1/*fliC*-P2, *hcpA*-P1/*hcpA*-P2, *tir*-P1/*tir*-P2, and *eae*-P1/*eae*-P2, respectively. The sizes of the gene fragments were 946 bp, 423 bp, 309 bp, and 811 bp, respectively. Restriction sites for four endonucleases (*Xho*I, *EcoR*I, *Sal*I, and *Xba*I) were incorporated into the PCR primers (**Table 2**). A linker sequence of “GCT GCTGCT AAA TTT GAT CAA ACC” was inserted between the *hcp*A gene, *tir* gene, and *eae* gene in order to separate the different domains [**13**]. The PCR products were treated with appropriate restriction enzymes, ligated, and cloned into Pcold I vector. The resulting plasmid was introduced into *E. coli* BL21 by chemical transformation according to the manufacturer’s instructions (pET System Manual, Novagen Company). Plasmids pET32-*fliC*, pET32-*hcp*A, pET32-*tir*, and pET32-*eae* were produced in a previous work. The primers and restriction enzymes are described in detail in **Table 2**. The pColdI-*fliC*-*hcp*A-*tir*-*eae* diagram is shown in **Fig. 1**.

**Figure 1:** Construction diagram of pCold I-*fli*C-*hcp*A-*tir*-*eae*. Four fragments of *fliC, hcpA, tir* and *eae* are amplified by PCR and ligated into pCold I by restriction enzyme. A linker sequence of “GCT GCTGCT AAA TTT GAT CAA ACC” is inserted between *hcp*A gene, *tir* gene and *eae* gene for more flexibility and efficient separation. Arrow shows the site of restriction enzyme.

**Table 2:** Primers.

primers	Sequence (5′–3′)^a^	Location in their ORF	Description
*fliC*-p1	ggggagctcactattaccaacaaa	538–1483 nt	5′ end of *fliC* with *Sac* I site
*fliC*-p2	ttactcgagggtcgttgcagaacc		3′ end of *fliC* with *Xho* I site
*hcp*A-p1	gggctcgagtttacacttatcgaactgat	19–441 nt	5′ end of *hcp*A with *Xho* I site
*hcp*A-p2	tttgaattc **tttagcagcagctttagcagcagc**gttggcgtcatc		3′ end of *hcp*A with *EcoR* I site
*tir*-p1	gatgaattcgagccggatagccca	775–1083 nt	5′ end of *tir* with *EcoR* I site
*tir*-p2	ttagtcgacagcccccgatgaaac		3′ end of *tir* with *Sal* I site
*eae*-p1	ttagtcgac **gctgctgctaaagctgctgctaaa**tttgatcaaacc	1995–2805 nt	5′ end of *eae* with *Sal* I site
*eae*-p2	ggctctagattattctacacaaaccgc		3′ end of *eae* with *Xba*I site

**a:** Unique restriction cleavage sites introduced in the oligonucleotides are underlined; linker sequences added to the primers are bold.

### Expression and Purification of Recombinant Protein

An overnight culture of *E. coli* BL21 (Pcold I-*fliC-hcpA*-*tir*-*eae*) was diluted 1∶50 into a flask each containing 200 mL LB broth. When bacteria were grown to the late exponential phase (OD600 = 1.2) at 37°C, the cultures were induced with 0.5 mM IPTG and incubated for additional 12 h at 15°C. The recombinant protein was purified according to the manufacturer’s instructions (Macherey-Nagel Corp.). The bacteria were pelleted by centrifugation at 12,000 *g* for 5 min and resuspended in 10 ml of 1×Lysis-Equilibration-Wash buffer (LEW) buffer. The concentrated bacterial suspensions were then sonicated (60% power, 5 s on, 5 s off, 10 min) and centrifuged at 12,000 *g* for 30 min again. The supernatant was collected and purified using His•Bind™ Resin Chromatography according to the manufacturer’s instructions (Macherey-Nagel Corp.). The expected size of recombinant His-H7-HCP-Tir-Intimin was approximately 88 kD. Similarly, recombinant Trx-H7, Trx-HCP, Trx-Tir, and Trx-Intimin proteins were expressed [**14]**–[**17**]. They were 51 kD, 34 kD, 30 kD, and 50 kD, respectively. The purity of these recombinant proteins was validated by SDS-PAGE and proteins were stored in −80°C (Figure 2).

**Figure 2:** The purity of Trx-H7, Trx-HCP, Trx-Tir, Trx-Intimin, and His-H7-HCP-Tir-Intimin was assayed by SDS-PAGE. Lane M, molecular mass standards; lane 1, His-H7-HCP-Tir-Intimin (88 kD); lane2, Trx-Intimin (50 kD);.lane 3, Trx-Tir (30 kD); lane 4, Trx-H7 (51 kD); lane 5, Trx-HCP (34 kD).

### Polyclonal Antibody Preparation and Western Blotting Assay

Specific polyclonal antibodies against His-H7-HCP-Tir-Intimin, Trx-H7, Trx-HCP, Trx-Tir, and Trx-Intimin were produced by subcutaneously injecting 4-month-old New Zealand white rabbits (2 rabbits per protein). Approximately 2 mL of recombinant vaccine containing 1 mg of purified protein was emulsified 1∶1 in Freund complete adjuvant was injected at multiple sites on the animals’ necks. The rabbits received one booster injection with the same amount of antigen emulsified 1∶1 with Freund’s incomplete adjuvant 21 days later. They were bled 10 days after the booster. Sera were filter (0.2 µm) sterilized and stored at −80°C until needed for a Western blotting assay.

The purified proteins were subjected to 12% SDS-PAGE and transferred to nitrocellulose membrane (Zhuyan Company, Nanjing). The membranes were blocked in 5% nonfat dry milk in Tris-Buffered Saline (TBS), pH 7.2, containing 0.1% Tween 20 (TBST) overnight at 4°C and then incubated with corresponding primary antibodies, including rabbit anti-H7, anti-HCP, anti-Tir and anti-Intimin (1∶1,000 dilution) for 2 h. After three washes with 0.5% nonfat dry milk in TBST, the membranes were incubated with a 1∶4,000 dilution of HRP-conjugated anti-rabbit IgG (Boster, Wuhan, China). Antigen-antibody complexes were visualized with the 3, 3′-diaminobenzidine (DAB) detection kit (Boster, Wuhan, China). Control immunoblots were performed with pre-immunization rabbit sera.

### Immunization and Challenge of Goats

Twelve 2-month-old male goats were divided into two groups and housed in 4 pens with three goats per pen. Goats were raised in the Animal House of Jiangsu Institute of Veterinary Medicine. On the day before vaccination (day 0), all animals were screened to confirm that they were negative for serum antibodies against His-H7-HCP-Tir-Intimin and that they did not shed *E. coli* O157:H7 in their feces. Six goats were injected subcutaneously at multiple sites on their necks with 200 µg/mL recombinant antigen emulsified1∶1(volume/volume) with ISA50V adjuvant (Seppic Company, France) on day 1, and given booster shots 3 weeks later. The remaining six goats were immunized with the same volume of ISA50V adjuvant. Serum samples and fecal samples were collected from all goats twice, on day 1 and again on day 35 (week 5).

Two weeks after the administration of booster shots, all goats were challenged orally with 10^9^ CFU *E. coli* O157:H7 strain 86-24 in 10 mL PBS using a drinking injector. Inoculation of each animal was completed within 2 min. Fecal excretion was monitored daily for two weeks, as described previously [**18**]. Briefly, each goat was hosted in a square cage (2 m×2 m) after challenge with *E. coli* O157:H7. Prior to fecal collection, a large piece of sterile gauze was placed under each cage. Fecal samples (10 g per animal) were collected on this sterile gauze in 10 mL PBS, softened by incubation with PBS for 2–4 h at 4°C and then homogenized in a stomacher. The homogenates were centrifuged at 500 *g* for 15 min to remove fecal materials. The supernatants were centrifuged at 11,000 *g* for 10 min, and the pellets were resuspended in 1 mL PBS followed by 10-fold serial dilutions. One hundred microliters of 10-fold dilutions were plated onto Sorbitol MacConkey (SMAC) agar plates containing novobiocin, tellurite, and vancomycin [**18]**–[**19**]. The remaining 900 µL of each dilution was enriched for 6 h at 41.5°C and subjected to the immunomagnetic bead separation (IMS) with O157 Dynabeads® (Invitrogen) according to the manufacturer’s instructions. After incubation, 100 µL was plated onto SMAC agar plates. Sorbitol-negative colonies were confirmed to be *E. coli* O157 with a latex agglutination test (Oxoid, Ltd., Basingstoke, U.K.). Duplex PCR of O157:H7 was performed according to the methods developed by our laboratory [**16**]. Colony counts were subjected to log 10 transformation for data analysis. If no colonies formed via direct plating, the concentration of *E. coli* O157 was set to 10 CFU/g by enrichment [**19]**–[**20**].

All the animals were euthanized 14 days after challenge using intravenous administration of 100 mg/Kg pentobarbital sodium. Then *E. coli* O157:H7 colonization was evaluated. Twenty-five grams of tissue from the rumen, abomasum, duodenum, jejunum, ileum, cecum, spiral colon, colon, rectum, and rectoanal junction (RAJ) of these experimental goats were collected. Tissue samples were homogenized using a stomacher and 10-fold serial dilutions were prepared. Tissue bacterial load was examined using direct culturing and IMS with O157 Dynabeads as described above in the description in the processing of feces.

### Determination of Serum IgG

Antibody responses specific to H7-HCP-Tir-Intimin were assessed using an enzyme-linked immunosorbent assay (ELISA) as described previously [**18]**–[**19**]. ELISA plates (Costar, U.S.) were coated with H7-HCP-Tir-Intimin protein (2.5 µg/mL in coating buffer) overnight at 4°C. The plates were blocked with 0.1% bovine serum albumin (BSA) in PBST. Two-fold serially diluted goat serum samples were added to the ELISA plates (100 µl/well) and incubated 1.5 h at 37°C. After washing three times with PBS containing 0.05% Tween 20 (PBST), rabbit anti-goat IgG-HRP (1/20,000 in PBST) (KPL Corporation) was added and incubated for 45 min at 37°C. Plates were washed 3 times with PBST, TMBS substrate solution (Sigma) was added to the mixture (100 µL/well) and incubated for 5 min at room temperature. The optical density (OD) at 450 nm was determined using a Sunrise™ Absorbance Reader (Sunrise, Austria). The titer was defined as the reciprocal of the highest dilution of a serum sample producing 2∶1 ratio value above the pre-immune level. Differences in immune responses between experimental groups were analyzed using Microsoft Excel and the t-test was used to evaluate antibody responses.

Western blot analysis was used to detect sera from vaccinated and naïve goats to confirm the results of the ELISA. Briefly, H7-HCP-Tir-Intimin protein resolved by PAGE was transferred to nitrocellulose and incubated with sera (1∶500 dilutions) from all experimental goats for 2 h each. Membranes were washed with TBST and incubated with a 1∶8,000 diluted rabbit anti-goat IgG-HRP (KPL Corporation). Immunoblots were visualized using a DAB detection kit (Boster, Wuhan, China).

Fecal ELISA was used to detect IgA in feces on day 1 and day 35. ELISA procedures were similar to those described above excepting that fecal samples and rabbit anti-goat IgA-HRP were used instead of goat sera and rabbit anti-goat IgG-HRP. Briefly, samples (approximately 5 g per animal) were mixed with 5 mL of PBS, vortexed until the pellets were not visible, and then centrifuged. The supernatant was 2-fold serially diluted in PBS and added to ELISA plates (100 µl/well). Rabbit anti-goat IgA-HRP (1/10,000 in PBST) (AbD Corporation) were used as the secondary antibody. To determine which component of H7-HCP-Tir-Intimin induces IgA secretion, additional ELISA assays were performed. In brief, plates (Costar, U.S.) were coated with Trx-H7, Trx-HCP, Trx-Tir, Trx-Intimin (2.5 µg/mL in coating buffer) overnight at 4°C. The remaining procedures were the same as what were described for fecal IgA ELISA. Differences in immune responses between experimental groups were analyzed using Microsoft Excel, and the t-test was used to analyze antibody responses.

### Bacterial Adherence to HEp-2 Cells

For adherence experiment, HEp-2 cells were cultivated at 37°C under 5% CO_2_ atmosphere in polystyrene 6-well plates (Costar,U.S) containing glass coverslips, as previously described [**20**]. For the adherence assay, cell monolayers at 70% confluency were washed and cultured with DMEM (Invitrogen). A sample (10 µl) of 2×10^7^ bacteria grown overnight in brain-heart infusion (BHI) plus NaHCO3 (BHIN) (Zhuyan Company, Nanjing,China) at 37°C was added to wells, and the cells were infected for 3 h, washed with PBS to remove unbound bacteria. Fresh medium was added to each well and incubated for additional 3 h and washed with PBS to remove the rest of unbound bacteria. Cells were fixed with 70% methanol/PBS for 5 minutes, and stained with Giemsa for 20 minutes. The coverslips were mounted on glass slides to be observed by light microscopy.

For experiment of suppressive adherence, the procedures were similar to those described above excepting that *E.coli* O157:H7 was incubated with vaccination sera before infection Hep-2 cells. Briefly, *E.coli* O157:H7 were mixed with 10-fold diluted vaccination sera and incubated at 37°C under 5% CO_2_ atmosphere for 30 min [**14**].

## Results

### SDS-PAGE and Western Blotting Analysis of Recombinant Proteins

All purified protein antigens were examined by SDS-PAGE and Coomassie blue staining. A single band of the expected molecular weight was identified for each protein sample (**Figure 2**). The H7-HCP-Tir-Intimin protein was detected in the supernatant fraction of lysed BL21 (Pcold I-*fliC-hcpA*-*tir*-*eae*), indicating the protein was soluble (**Figure 3A**). To determine whether each component of recombinant H7-HCP-Tir-Intimin protein was immunogenic, Western blot analyses were carried out using rabbit anti-H7, anti-HCP, anti-Tir, and anti-Intimin sera, with pre-immunization sera as a negative control. Results showed that recombinant H7-HCP-Tir-Intimin protein reacted strongly to these-mentioned sera, as evidenced by the distinct band for each corresponding antibody and the lack of reactivity to pre-immunization sera (**Figure 3B**). The data indicated that each component of H7-HCP-Tir-Intimin had strong immunogenicity.

**Figure 3:** His-H7-HCP-Tir-Intimin was assayed by SAS-PAGE and Western blot. A: Lane 1, BL21 (Pcold I-*fliC-hcpA*-*tir*-*eae*) uninduced. Lane 2 shows the precipitation of BL21 (Pcold I-*fliC-hcpA*-*tir*-*eae*) induced by IPTG; lane 3 BL21 (Pcold I-*fliC-hcpA*-*tir*-*eae*) supernatant. Lane M protein marker. B: Purified His-H7-HCP-Tir-Intimin was identified using rabbit anti-H7, anti-HCP, anti-Tir, anti-Intimin, and pre-immunization sera. Lanes 1–5, purified His-H7-HCP-Tir-Intimin; lanes 6–10, immunoblots with anti-H7, anti-HCP, anti-Tir, anti-Intimin, and pre-immunization sera.

### Stimulation of Immune Responses in Subcutaneously Immunized Goats

On day 7, vaccinated goats produced an average IgG titer of 733. Specifically, 4 vaccinated goats had IgG titers of 800 and the remaining 2 goats had titers of 200 and 1600, respectively (**Figure 4A**). On day 21, the immunized goats had an average titer of 1.4×10^5^. The average IgG titer peaked after administration of booster shots (day 35) containing H7-HCP-Tir-Intimin, at 7.2×10^5^ (**Figure 4B**). Each serum sample was then further evaluated by Western blot analysis. The present results indicate that vaccination sera interacted with recombinant H7-HCP-Tir-Intimin protein, and naïve sera did not.

**Figure 4:** ELISA of H7-HCP-Tir-Intimin–specific IgG titers of sera from immunized and non-immunized subjects. Blood was sampled from all goats at 0 d, 21 d, and 35 d (14 d post-booster) to determine IgG titers (A and B). A: Each immunized goat and naïve goat. 1–6: immunized goats; 7–12: naïve goats. The immunization induced IgG at 7 d, and this effect increased distinctly at 21 d (*P* = 0.0030) and immediately after the booster (*P* = 0.0166), but the naïve goats showed no such IgG reactions. B: Statistical analysis of average IgG titer of vaccinated goats.

In addition, secretory IgA titers specific for H7-HCP-Tir-Intimin, H7, HCP, Tir and Intimin were determined using ELISA. Two weeks after the booster shot, H7-HCP-Tir-Intimin-specific IgA was detected in the feces of 5 goats, H7-specific IgA was detected in 4 goats, HCP-specific IgA was detected in 5 goats, and no IgA was detected in any of the unvaccinated animals. These results suggest that H7 and HCP of H7-HCP-Tir-Intimin antigen play a vital role in eliciting IgA secretion into the intestinal lumen (**Figure 5**).

**Figure 5:** ELISA for H7-HCP-Tir-Intimin specific IgA titers of feces in immunized goats. Fecal samples were taken from all goats at 0 d and 35 d (14 d post-booster) to test IgA titers. Five vaccinated goats secreted high titers of HCP- and H7-HCP-Tir-Intimin-specific IgA in feces, four animals produced certain titers of H7-specific IgA. The remaining samples, not shown here, showed no results.

### Challenge and Excretion of *E. coli* O157:H7

After challenge with *E. coli* O157:H7, no goats developed diarrhea. Vaccinated animals shed significantly less bacteria than goats of the placebo group (*P* = 0.0109) (**Figure 6**). From day 5 on, *E. coli* O157:H7 was not detected in the feces of vaccinated goats. One vaccinated goat stopped shedding on day 3. In contrast, all but one of the naïve animals shed bacteria throughout the course of challenge (14 days). That goat became negative on day 10.

**Figure 6:** *E. coli* O157:H7 shedding in feces after subcutaneous administration in goats. Two weeks after secondary immunization, all goats in both groups were fed 10^9^ CFU O157:H7 and fecal shedding was monitored every day for two weeks. The error bar shows the standard deviation and differences in outcome were assessed using a t-test (*P* = 0.0109).

After euthanasia, direct fecal culture was positive for 5 naive animals. *E. coli* O157:H7 carriage in feces ranged from 5.6×10^4^ CFU/g to 3.2×10^2^ CFU/g. After the enrichment and IMS, all intestinal tissues of the placebo-vaccinated animal were positive, but *E. coli* O157:H7 was not found in any vaccinated animals, indicating that tissue colonization was minimal or undetectable.

### Bacterial Adherence to HEp-2 Cells

To further evaluate the significance of H7-HCP-Tir-Intimin antibody, each goat serum sample was detected *in vitro* by HEp-2 cells. For infection experiments, we propagated *E.coli* O157:H7 overnight in BHIN at 37°C in order to advance adherence. The light microscopy images of infected, Giemsa-stained cells showed obvious impairment of adherence of *E.coli* O157:H7 after incubation with vaccination sera as compared with naive sera (**Figure 7**).

**Figure 7:** Optical microscopy analysis of suppressive adherence of *E.coli* O157:H7 to HEp-2 cells by vaccination sera from goats. **A:** *E.coli* O157:H7; **B:** *E.coli* O157:H7 incubated with naive sera; **C–H:** *E.coli* O157:H7 incubated with vaccination sera from each goat. Red arrow represents bacteria, green arrow represents cells. Magnifications, ×400.

## Discussion

In the present study, a goat model was used to evaluate the efficacy of a recombinant H7-HCP-Tir-Intimin vaccine on *E. coli* O157:H7 fecal shedding and host immune responses after exposure. Strong evidence showed that H7-HCP-Tir-Intimin could significantly reduce fecal shedding and provoke specific immune responses.

Because small ruminants are potential reservoirs of *E. coli* O157:H7, effective vaccines for these host species will have important significance to public health. In the present study, the majority of the naïve goats, all but one, shed *E. coli* O157:H7 throughout the entire detection period. All the tissues of their intestinal tracts were positive for *E. coli* O157:H7. This is consistent with previous reports stating that 8-week-old conventionally reared goats inoculated orally with *E. coli* O157:H7 shed bacteria until the 18^th^ day after inoculation [**21**]. Animals examined on day 4 after inoculation showed multifocal AE lesions in the distal colon, rectum, and at the recto-anal junction [**21**]. Another study demonstrated that an 8-week-old goat kid fed *E. coli* O157:H7 shed the bacteria in large numbers. These numbers increased upon coincidental *C. parvum* infection [**22**]. One report showed that 20 people became ill and 1 died from *E. coli* O157 in organic goat’s milk cheese has been published online (http://barfblog.com/2013/09/20-sick-1-dead-from-e-coli-o157-in-raw-milk-organic-goats-milk-cheese-columnist-says-dont-overreact/.) One report on an *E. coli* O157 outbreak in Scotland was linked to unpasteurized goat’s milk has been published online (http://www.eurosurveillance.org/ViewArticle.aspx?ArticleId=1387). In Greece, *E. coli* serogroup O157 was used to isolate of 24 strains (1.4%) of which 21 were isolated from bovine milk (2.2%) and 3 from caprine milk (0.7%) [**23**]. A study performed in Switzerland indicated that 16.3% of the evaluated goats’ milk and 12.7% of ewes’ milk were PCR-positive for Shiga-toxin-producing *E. coli* [**24**]. To date, there have been several investigations focusing on vaccine development aimed at preventing the shedding of *E. coli* O157:H7. A vaccine based on the translocon proteins EspA and EspB, and Intimin significantly reduced fecal shedding of *E. coli* O157:H7 in orally infected sheep [**25**]. Intranasal immunization with Stx2B-Tir-Stx1B-Zot protein led to less shedding in goats after experimental infection with *E. coli* O157:H7 [**18**]. The results of these studies confirmed that vaccination of small ruminants with recombinant subunit vaccines can reduce the *E. coli* O157:H7 burden in goats.

The development of multi-component vaccines has become a priority of modern vaccine research. In the current study, a tetravalent recombinant vaccine (H7-HCP-Tir-Intimin) comprising the central region of H7 (H7315), nearly full-length HcpA (HcpA141), the carboxy terminus of Intimin (Intimin270), and the exposed C-end region of Tir (Tir103) was constructed and evaluated. H7 and HCP were chosen because these proteins can block bacterial attachment in the early stage of colonization. Tir is an important T3SS protein. It acts as a receptor for Intimin. Both Tir and Intimin are the preferred choices for recombinant subunit vaccines. In cattle, vaccination with supernatant preparations containing T3SS proteins does decrease *E. coli* O157:H7 shedding in naturally infected steer [**4**]. A benefit to using supernatant proteins is that the preparation contains not only T3SS proteins but also flagellin, HCP, and lipopolysaccharide (LPS), which contribute to the efficacy of the vaccine. For this reason, flagellin and HCP should be selected as essential components to construct subunit vaccines.

The data from the current study showed that recombinant H7-HCP-Tir-Intimin can prevent *E. coli* O157 colonization in goats. After the initial inoculation, serum IgG titers increased significantly. In order to improve immune responses, a booster was administered three weeks after primary immunization, the same schedule used for cattle vaccines prepared from the supernatant of bacterial cultures for achieve optimal immunity [**4]**, [**26**]. In the present study, the IgG titer against H7-HCP-Tir-Intimin increased 3 times after booster (7.2×10^5^) compared to the titer at the primary immunization (1.4×10^5^). Western blotting was carried out to assess host immune responses, and each serum from all vaccinated goats reacted to H7-HCP-Tir-Intimin, confirming the immunogenicity of the recombinant protein. Experiment of suppressive adherence to HEp-2 cells was used to evaluate the blocking ability of H7-HCP-Tir-Intimin antibody, and each serum from all vaccinated goats reduced the number of adherent bacteria to HEp-2 cells.

Fecal shedding is an important parameter of the effectiveness of recombinant *E. coli* O157:H7 antigens [**4]**–[**7**]. Our data showed there to be significantly less fecal shedding of *E. coli* in vaccinated goats than in control animals (*P* = 0.0109) (**Figure 6**). *E. coli* O157:H7 was not detected in the feces of any vaccinated goats at any point after day 5. In contrast, most naïve goats shed bacteria throughout the course of the challenge (14 days). McNeilly et al. demonstrated that intramuscular vaccination with a combination of intimin-531, the translocon filament protein, EspA, Tir, and H7 flagellin significantly reduced shedding of *E. coli* O157 from experimentally infected cattle [**7**]. However, no study has yet shown whether goats vaccinated with this vaccine shed less *E. coli* O157:H7. The vaccine discussed in this paper included four immunogens, but they were expressed separately and then mixed to prepare the vaccine. This way of preparing vaccine is not economically efficient or convenient. A better vaccine design in our study is to prevent both the first adherence of *E. coli* O157:H7 and the consequent invasion into epithelial cells using animal immunization. For this reason, HCP and H7 were used to block initial adherence and intimin and Tir were used to block invasion and colonization. In order to prepare the vaccine more easily, all individual genes were linked to the same vector of Pcold I to express one protein, in this case H7-HCP-Tir-Intimin. This plasmid vector can be used to express soluble proteins in a manner similar to their natural form [**Cat.# 3360–3364, TaKaRa Corp.**]. Whether the tetravalent vaccine provides the same efficacy in cattle remains to be proven. Cattle experiments must be designed to confirm its effectiveness. In summary, the tetravalent recombinant H7-HCP-Tir-Intimin vaccine was here found to prevent *E. coli* O157:H7 intestinal colonization and fecal shedding.

Present data also show that H7 flagella and HCP play important roles in mitigating bacterial shedding and persistence in the goat intestinal tract. Flagellin has been proposed as a vaccine candidate because of its intrinsic adjuvant activity, which is mediated through TLR5 [**27]**–[**28**]. Recent findings, however, suggest that vaccines against flagellated pathogens should avoid inducing antibodies (Abs) against TLR5 because antibody production may help flagellated bacteria evade host clearance by reducing the host’s ability to mount an innate immune response [**28]**–[**30**]. The NH2- and COOH-terminal regions of flagellin are involved in interactions with TLR5 and are well conserved among various Gram-negative bacteria [**30**]. To circumvent this problem, the regions responsible for interacting with TLR5 were removed during the construction of the H7-HCP-Tir-Intimin tetra-protein. The results proved that H7-HCP-Tir-Intimin could prevent bacterial colonization. In contrast, a previous study showed that systemic immunization of calves with full H7 flagellin only delayed peak bacterial shedding, by approximately 1 week [**9]**, [**27**]. In the present study, most vaccinated goats had detectable H7 specific-IgA in their feces with titers ranging from 2 to 16. The present results are consistent with the findings reported by McNeilly et al. [**9**]. HCP, a novel virulence factor of *E. coli* O157:H7, was shown to be involved in bacterial adherence, invasion, hemagglutination, biofilm formation, twitching motility, and extracellular matrix glycoprotein binding [**10]**–[**11**]. In the present study, H7-HCP-Tir-Intimin vaccination elicited high titers of HCP-specific IgA in most goats. A previous study showed that recombinant HCP induced the production of specific IgG and IgA and impaired *E. coli* O157:H7 colonization in the mouse gut [**15**]. Taken together, the central region of H7 flagellin and full-length HCP could be important functional components of the recombinant tetra unit protein during blockage of bacterial colonization.

It has been reported that culture conditions play an important role in the ability of EHEC O157:H7 to adhere to cultured cells and to epithelial cells in the pig terminal ileum [**31**]. Also, the maturation of a functional TTSS is accelerated in EHEC O157:H7 by restricting the concentration of oxygen [**32**]. Bicarbonate ions can activate expression of LEE and certain non-LEE encoded genes, resulting in greater adherence of EHEC O157:H7 *in vitro* and increased shedding from 14-week-old pigs [**33]**–[**34**]. To ensure the success of goat challenge, *E. coli* O157:H7 was cultured in brain-heart infusion (BHI) plus NaHCO3 (BHIN) with gentle shaking. There were more bacteria adhering to HEp-2 under these conditions than in LB with vigorous shaking (data not shown). Collectively, the use of cultural conditions mimicking *in vivo* environment is essential to the development of a successful animal model for the evaluation of vaccines.

In conclusion, vaccination of goats with recombinant H7-HCP-Tir-Intimin protein reduced fecal shedding of EHEC O157:H7 very effectively. The recombinant protein can be easily produced in large quantities and the production can be standardized for consistent performance. Data from the current investigation warrants further clinical trials aimed at reducing bacterial load on farms and mitigating the contamination of carcasses by EHEC O157:H7.
